# Risk of visual impairment according to the comorbidity of systemic and ocular diseases

**DOI:** 10.1371/journal.pone.0307011

**Published:** 2024-09-05

**Authors:** Juwon Choi, Youn Joo Choi, Kyoung Lae Kim, Yong-Kyu Kim, Sung Pyo Park, Kyeong Ik Na

**Affiliations:** Department of Ophthalmology, Kangdong Sacred Heart Hospital, Hallym University College of Medicine, Seoul, Korea; Hangil Eye Hospital / Catholic Kwandong University College of Medicine, REPUBLIC OF KOREA

## Abstract

**Purpose:**

To investigate the risk of visual impairment (VI) based on the presence or absence of four diseases: hypertension (HTN), diabetes mellitus (DM), glaucoma, and diabetic retinopathy (DR).

**Methods:**

This retrospective population-based study included 1,000,000 randomly selected participants from the National Health Checkup Program database between 2015 and 2016. VI was defined as a presenting visual acuity ≤ 0.5 in the better eye. The participants were divided into 12 groups according to the presence or absence of disease. Adjusting for age and sex, the risk of VI in each disease group was analyzed and compared with the others.

**Results:**

Among the 1,000,000 participants, 88,931 (8.89%) had VI. The odds ratios (ORs) of age, male sex, HTN, DM, glaucoma, and DR for VI were 1.06 (95% CI, 1.05–1.06), 0.52 (95% CI, 0.52–0.53), 1.11 (95% CI, 1.09–1.13), 1.07 (95% CI, 1.05–1.09), 0.92 (95% CI, 0.90–0.74), and 1.29 (95% CI, 1.25–1.34), respectively (all *P* < 0.001). The group with HTN, DM, glaucoma, and DR had the highest OR of 1.98 (*P* < 0.001) compared to the healthy group. HTN, DM, and DR were positively correlated with VI in all groups. Glaucoma was positively correlated in the group with DM and DR and in the group with HTN, DM, and DR (ORs 1.18, 1.11, all *P* < 0.05); however, it demonstrated a negative correlation in the other groups (ORs 0.85–0.93, all *P* < 0.05).

**Conclusion:**

HTN, DM, and DR, either alone or in combination, increase the risk of VI. Glaucoma also increases the risk when combined with DR; however, it has a negative correlation with VI in the absence of DR. Periodic ophthalmologic examinations for glaucoma, which primarily affects the peripheral visual field and not central visual acuity, might help prevent VI caused by other diseases.

## Introduction

Vision is one of the most important physical factors affecting quality of life. Furthermore, in older age, visual impairment (VI) not only significantly affects quality of life [1,2] but also amplifies comorbidities such as cognitive impairment [3] and risk of falls [4,5]. VI also has socioeconomic repercussions, such as an increase in social costs and a decrease in productivity [6–10].

The estimated number of individuals living with VI globally is 285 million, of whom 39 million are blind and 246 million have low vision [11]. The principal causes of VI include under-corrected refractive errors, cataracts, glaucoma, age-related macular degeneration, myopic macular degeneration, and diabetic retinopathy (DR) [4,11–15]. Additionally, certain chronic systemic adult diseases such as diabetes mellitus (DM) and hypertension (HTN) are considered risk factors for VI [16–18].

Previous studies have mainly focused on the relationship between a single disease and VI and elucidated the effects of some closely related diseases (such as DM and DR) on visual acuity [12,13,19–23]. To the best of our knowledge, no study has examined how the risk of VI differs according to the combination of several diseases.

Hence, we decided to analyze the risk of VI according to the presence or absence of HTN, DM, glaucoma, and DR using the National Health Checkup Program data and the claims data of each disease. We also investigated the effect of each disease on VI in combination with other diseases.

## Materials and methods

This study is retrospective design and only anonymized data were obtained, it has been approved an exemption by the Institutional Review Board of the Kangdong Sacred Heart Hospital (KANGDONG 2022-07-001) and adheres to the ethical principles outlined in the Declaration of Helsinki.

### National health checkup program

The National Health Checkup Program is a nationwide program conducted by the National Health Insurance Service (NHIS). This program targets the Korean population and requires the mandatory participation of eligible individuals. The National Health Checkup Program is conducted at NHIS-certified hospitals once every 2 years and includes employed subscribers of all ages, local household heads, and household members aged 40 years and older who are insured [24]. As part of this program, trained examiners measure participants’ height, weight, hearing, and visual acuity, and conduct laboratory tests as well.

### Study population

We analyzed the data randomly extracted 1,000,000 individual records from the National Health Checkup Program database between 2015 and 2016. The data were released to the public by the NHIS [25] and included age, sex, visual acuity, and presence or absence of four diseases; HTN, DM, glaucoma, and DR. If the participant had a claim record with the disease code in the NHIS database, he/she was considered to have the disease. Each disease code was as follows: HTN (I10-I13, I15), DM (E10-E14), glaucoma (H40, H42), and DR (E10.31-E10.33, E11.31-E11.33, E12.31-E12.33, E13.31-E13.33, E14.31-E14.33, H360). The received data were all de-identified.

### Definition of visual impairment

Presenting visual acuity was measured by the National Health Check-up Program. Presenting visual acuity is the uncorrected visual acuity of those who do not wear corrective spectacles or the corrected visual acuity of those who wear spectacles in their daily life [26]. The visual acuity data were recorded as values ranging from 0.1 to 2.5. If the visual acuity was less than 0.1, it was recorded as 0.1. In our study, we defined VI as a presenting visual acuity of 0.5 or less in the better eye, referencing the United States criteria, where low vision is defined as a best-corrected visual acuity less than 20/40 in the better eye.

### Classification of disease groups

The participants were divided into the following 12 groups according to the presence or absence of each disease: Healthy, group without HTN, DM, glaucoma, or DR; H, group with only HTN; D, group with only DM; G, group with only glaucoma; HD, group with HTN and DM; HG, group with HTN and glaucoma; DG, group with DM and glaucoma; D_R, group with DM and DR; HDG, group with HTN, DM, and glaucoma; HDR, group with HTN, DM, and DR; DGR, group with DM, glaucoma, and DR; and HDGR, group with HTN, DM, glaucoma, and DR.

### Statistical analysis

Age, sex, and disease status were compared between the VI and control groups using the t-test for continuous variables and the chi-square test for categorical variables. Multiple logistic regression analyses were used to determine the odds ratios (ORs) for VI based on age, sex, and disease status. To evaluate the risk of VI in each disease group compared to the other disease groups, the OR of each disease group was analyzed by setting all other groups as a reference group and adjusting for age and sex in multiple logistic regression analyses. Additionally, we conducted these analyses separately by dividing the participants into the following three age groups: 20–39 years, 40–59 years, and 60 years and above.

All statistical analyses were performed using the open-source R software package version 4.0.3 (R Project for Statistical Computing, Vienna, Austria). Statistical significance was considered as a *p*-value less than 0.05.

## Results

The total number of participants with VI was 88,931 out of 1,000,000, and the prevalence of VI was 8.89%. (Table 1) The mean ages of the VI and control groups were 58.4±15.4 and 47.7±13.6 years (*P* < 0.001), respectively. Men comprised 34.9% of the VI group and 52.5% of the control group (*P* < 0.001). In the VI group, the prevalences of HTN, DM, glaucoma, and DR were 44.4%, 25.4%, 17.3%, and 5.7%, respectively, which were significantly higher than those in the control group (25.4%, 14.5%, 13.6%, and 2.4%, respectively; all *P* < 0.001).

**Table 1:** Demographic characteristics and prevalence of diseases in the visual impairment and control groups.

	All			20–39 years group			40–59 years group			60 years group		
	VI	Control	*P-value* *	VI	Control	*P-value* *	VI	Control	*P-value* *	VI	Control	*P-value* *
Number	88,931	911,069		13,145	286,872		29,030	454,372		46,756	169,825	
Age (yrs)	58.4±15.4	47.7±13.6	<0.001	30.5±5.9	32.0±5.7	<0.001	51.5±5.7	50.2±5.7	<0.001	70.6±4.9	67.7±4.9	<0.001
Men (%)	34.9	52.5	<0.001	42.5	57.9	<0.001	32.7	50.3	<0.001	34.1	49.2	<0.001
HTN (%)	44.4	25.4	<0.001	3.5	4.6	<0.001	28.8	25.6	<0.001	65.6	60.2	<0.001
DM (%)	25.4	14.5	<0.001	3.4	2.9	0.001	18.6	14.5	<0.001	35.8	33.9	<0.001
Glaucoma (%)	17.3	13.6	<0.001	8.3	8.4	0.715	15.0	13.5	<0.001	21.2	22.5	<0.001
DR (%)	5.7	2.4	<0.001	0.5	0.3	<0.001	4.2	2.2	<0.001	8.1	6.9	<0.001

VI, visual impairment; HTN, hypertension; DM, diabetes mellitus; DR, diabetic retinopathy.

* *The p*-values were calculated using an independent t-test for continuous variables and a chi-square test for categorical variables.

In the multivariate analysis, VI was positively associated with older age (OR 1.06, 95% confidence interval [95% CI] 1.05–1.06, *P* < 0.001), HTN (OR 1.11, 95% CI 1.09–1.13, *P* < 0.001), DM (OR 1.07, 95% CI 1.05–1.09, *P* < 0.001), and DR (OR 1.29, 95% CI 1.25–1.34, *P* < 0.001) (Table 2). VI was negatively associated with male sex (OR 0.52, 95% CI 0.52–0.53, *P* < 0.001) and glaucoma (OR 0.92, 95% CI 0.90–0.94, *P* < 0.001).

**Table 2:** Multiple logistic regression analysis for age, sex, and disease status in the visual impairment group, using the control group as a reference.

	All		20–39 years group		40–59 years group		60 years group	
	Odds ratio	*P-value*	Odds ratio	*P-value*	Odds ratio	*P-value*	Odds ratio	*P-value*
Age	1.06 (1.05–1.06)	<0.001	0.96 (0.96–0.96)	<0.001	1.04 (1.03–1.04)	<0.001	1.13 (1.12–1.13)	<0.001
Men	0.52 (0.52–0.53)	<0.001	0.55 (0.53–0.57)	<0.001	0.47 (0.46–0.49)	<0.001	0.54 (0.52–0.55)	<0.001
HTN	1.11 (1.09–1.13)	<0.001	0.94 (0.86–1.04)	0.240	1.07 (1.04–1.10)	<0.001	1.00 (0.98–1.02)	0.938
DM	1.07 (1.05–1.09)	<0.001	1.36 (1.22–1.51)	<0.001	1.18 (1.14–1.22)	<0.001	0.98 (0.95–1.00)	0.075
Glaucoma	0.92 (0.90–0.94)	<0.001	0.93 (0.88–1.00)	0.036	1.01 (0.97–1.04)	0.634	0.83 (0.81–0.85)	<0.001
DR	1.29 (1.25–1.34)	<0.001	1.66 (1.25–2.19)	<0.001	1.65 (1.54–1.77)	<0.001	1.19 (1.14–1.24)	<0.001

HTN, hypertension; DM, diabetes mellitus; DR, diabetic retinopathy.

Out of the 1,000,000 participants, 594,305 (59.4%) were classified into the healthy group and had no HTN, DM, glaucoma, or DR (Table 3). By contrast, 6,610 (0.66%) participants had all four diseases and were accordingly categorized into the HDGR group. Including the above two groups, the study participants were divided into 12 groups according to the presence or absence of diseases.

**Table 3:** Number of participants in each disease group.

Disease group	All	20–39 years group	40–59 years group	60 years group
Healthy	594,305	256,964	284,823	52,518
H___	146,069	10,240	74,885	60,944
_D__	41,859	5,253	24,619	11,987
__G_	74,874	22,910	39,782	12,182
HD__	60,983	1,848	25,912	33,223
H_G_	30,367	1,081	12,701	16,585
_DG_	8,795	657	4,696	3,442
_D_R	5,973	386	3,229	2,358
HDG_	15,440	220	4,940	10,280
HD_R	11,856	178	4,227	7,451
_DGR	2,869	195	1,448	1,226
HDGR	6,610	85	2,140	4,385

Healthy, group without HTN, DM, glaucoma, or DR; H, group with only HTN; D, group with only DM; G, group with only glaucoma; HD, group with HTN and DM; HG, group with HTN and glaucoma; DG, group with DM and glaucoma; D_R, group with DM and DR; HDG, group with HTN, DM, and glaucoma; HDR, group with HTN, DM, and DR; DGR, group with DM, glaucoma, and DR; HDGR, group with HTN, DM, glaucoma, and DR.

Each disease group was compared with the other groups as references to estimate the risk of VI. Among 132 multiple logistic regression analyses adjusted for age and sex, 122 were significant. The HDGR group, compared to the healthy group, had the highest OR of 1.98 (95% CI 1.86–2.11, *P* < 0.001) and followed by the HDGR group, compared to the G group (OR 1.94, 95% CI 1.81–2.08, *P* < 0.001) (Fig 1).

**Fig 1:** Odds ratios for visual impairment of each disease group using the other disease groups as reference groups. Multiple logistic regression analysis results where the *P*-value is less than 0.05 are marked; otherwise, the results are marked as blank.

In the 20–39 years age group, 57 analyses were significant. The DGR group, compared to the HG group, had the highest ORs of 3.31 (95% CI 1.86–5.89, *P* < 0.001), followed by the DGR group, compared to the H group (OR 3.20, 95% CI 1.99–5.15, *P* < 0.001) (Fig 2).

**Fig 2:** Odds ratios for visual impairment of each disease group using the other disease groups as reference groups in the 20–39 years age group.

In the 40–59 years age group, 102 analyses were significant. The HDGR group, compared to the G group, had the highest OR of 2.96 (95% CI 2.60–3.38, *P* < 0.001), followed by the HDGR group, compared to the healthy group (OR 2.83, 95% CI 2.50–3.19, *P* < 0.001) (Fig 3).

**Fig 3:** Odds ratios for visual impairment of each disease group using the other disease groups as reference groups in the 40–59 years age group.

In the 60 years and older group, 90 analyses were significant. The DGR group, compared to the DG group, had the highest OR of 1.47 (95% CI 1.25–1.73, *P* < 0.001), followed by the HDGR group, compared to the DG group (OR 1.45, 95% CI 1.30–1.63, *P* < 0.001) (Fig 4).

**Fig 4:** Odds ratios for visual impairment of each disease group using the other disease groups as reference groups in the 60 years and older age group.

The comparative analysis results of the disease groups with and without a specific disease were separated to visualize the OR of that specific disease for VI (Fig 5). For instance, we aimed to investigate how the risk of VI changed when HTN was added to each disease group by pooling the multiple logistic regression results of the H and healthy, HD and D, HG and G, HDG and DG, HDR and DR, and HDGR and DGR groups.

**Fig 5:** Odds ratios for visual impairment of each disease in the different disease groups.

HTN was positively correlated with VI in all disease groups when it was added. These correlations were significant in all groups except the D group. DM was positively correlated with VI in all disease groups. These correlations were significant in both the healthy and G groups. DR showed significant positive correlations with VI in all disease groups. Glaucoma was positively correlated with VI in the D_R and HDR groups, whereas it was negatively correlated with VI in the healthy, H, D, and HD groups. These correlations were significant in all the groups.

## Discussion

In this population-based study, the prevalence of VI was 8.9% among those aged 20 years and older. Additionally, among those aged 40 years and older, the prevalence was 10.8%. Previous studies have reported the prevalence of VI, which is defined as presenting visual acuity of 0.5 or less in the better eye [21,22]. The Singapore Indian Eye Study reported a prevalence of 16.8% for VI in ethnic Indians aged 40 years and older living in Singapore [22]. The Taizhou Eye Study reported a prevalence of 18.2% for low vision and 1.9% for blindness in the Chinese population aged 45 years and older [21]. The lower prevalence of VI observed in this study compared to that in previous studies can be attributed to differences in the study populations and the potential influence of recent widespread corneal refractive surgeries in Korea. In this study, similar to previous studies, male sex was negatively correlated with VI [21].

In this study, the OR for VI in patients with HTN was 1.11 (95% CI 1.09–1.13, *P* < 0.001). These results show that HTN is positively correlated with VI and increases the risk of various vision-threatening conditions that affect ocular structure and function. HTN is also an important risk factor for the development of blinding vascular diseases, such as retinal vein and artery occlusion, emboli in retinal arterioles, and DR [27,28]. However, HTN did not show a significant association with VI in the 20–39 years and the 60 years and older age groups in this study. Conversely, HTN was significantly associated with VI in the 40–59 years age group. We speculate that the lack of a significant association between HTN and VI in the 20–39 years age group may be due to the relatively short duration of illness in this group. Conversely, in the 40–59 years age group, as the duration of hypertension increased, the likelihood of HTN affecting vision increased, resulting in a significant association between HTN and VI. However, in the 60 years and older age group, it is believed that the influence of other age-related conditions, such as cataracts and macular degeneration on vision, became stronger, leading to a relatively weaker association between HTN and VI [29]. In a previous study, HTN did not show a significant association with VI (OR 1.74, 95% CI 0.87–3.51, *P* = 0.120) in a multiple regression analysis of data collected from Eastern Taiwanese participants aged 55 years and older [16].

In this study, the OR of DM for VI was 1.36 (95% CI 1.22–1.51, *P* < 0.001) in the 20–39 years age group, which was higher than that in the 40–59 years age group with an OR of 1.18 (95% CI 1.14–1.22, *P* < 0.001), and not significant in the 60 years and older age group with an OR of 0.98 (95% CI 0.95–1.00, *P* = 0.075). This suggests that younger patients with DM are at a higher risk of developing VI. Zhang et al. reported that the difference in correctable VI between individuals with and without DM was greatest in the younger age group [30]. Similar to our study, Wang et al. reported no significant association between DM and VI based on an analysis of participants aged 55 years and older [16]. However, DR showed a significant positive correlation with VI in all participants and across all age groups in our study. Zeried et al. reported the OR for VI in patients with DR as 1.22 (95% CI 1.05–1.95, *P* = 0.04) in participants aged 40 years and older [29].

Glaucoma is one of the most common causes of irreversible blindness. Glaucoma was ranked as the second leading cause of blindness and the fourth leading cause of moderate and severe VI in a global analysis [31]. However, the OR for VI in patients with glaucoma was 0.92 (95% CI 0.90–0.94, *P* < 0.001) in our study, which was less than 1, indicating a negative correlation between glaucoma and VI. Therefore, we analyzed the data to determine the effect of each disease on VI by dividing the participants into several groups according to the presence or absence of each disease, including glaucoma.

We analyzed and compared the ORs for VI across the different disease groups, and significant results were observed in 122 of the 132 analyses. In the age-stratified analysis conducted with three age groups, the 20–39 years group showed significant results in 57 analyses, less than those in the older age groups of 40–59 and 60 years and older (102 and 90 analyses, respectively). By contrast, the highest ORs observed in the 20–39, 40–59, and 60 years and older groups were 3.31, 2.96, and 1.47, respectively, indicating a higher OR for VI in the younger age groups. This indicates that the risk of VI increases rapidly when multiple diseases coexist, particularly among younger individuals.

Compared with the healthy group, in the HDGR group the OR for VI was 1.98, indicating that an individual with HTN, DM, glaucoma, and DR has a 1.98 times higher risk of VI than a healthy person. It is a convincing result when considering the relationship between these diseases and VI. Moreover, a noteworthy point is that the G group showed a negative correlation with VI when compared to the other groups, even when compared to the healthy group.

In the 20–39 years age group, the ORs for VI in the DGR group were the highest in all analyses. In other words, the coexistence of glaucoma and DR in the younger age group had a significant effect on visual acuity. It is reported that in the 20–39 years group, those who have been suffering from DM for 10 years or more are more likely to have type 1 DM, and the risk of VI is greater than that of type 2 DM [32]. Type 1 DM carries a 5.94 times higher risk of secondary glaucoma, such as neovascular glaucoma, than type 2 DM [33]. We thought that these findings explain the high risk of VI observed in the DGR group in the 20–39 years age group.

In the 40–59 years age group, 102 of 132 analyses showed a significant result, which was a greater number than that in the 20–30 years age group. However, in the 60 years and older age group, the number of significant results decreased to 90 of 132 analyses. Furthermore, there was a tendency for the OR to decrease as age increased. This means that the effects of HTN, DM, glaucoma, and DR on visual acuity decreased in the 60 years and older age group compared to those in the 40–59 years group. This suggests that other factors that affect visual acuity, such as macular degeneration and cataracts, play a greater role with age [11–15]. In addition, in the 60 years and older age group, it showed a different pattern in the 20–39 years and 40–59 years age groups. Compared with most other groups, the glaucoma group without DR exhibited a negative correlation with VI.

To further clarify the association between glaucoma and VI, we evaluated the impact of each disease on VI. A comparison of the pairs of groups with and without a specific disease is summarized in Fig 5. HTN, DM, and DR were positively correlated with VI in all groups, and these results were significant in most groups. Glaucoma showed a significant positive correlation with VI when coexisting with DR; however, it showed a significant negative correlation when not accompanied by comorbid DR.

Glaucoma causes gradual peripheral vision loss, which can progress to tunnel vision in advanced stages; however, it has relatively little effect on visual acuity in the earlier stages. Moreover, glaucoma requires regular monitoring for progression. Owing to these characteristics, patients with glaucoma can proactively prevent, detect, and treat various conditions that can impair vision before VI occurs through regular ophthalmologic examinations. In addition, patients diagnosed with glaucoma may be sensitive to changes in their visual acuity, which can also have an impact. However, in cases where glaucoma coexists with DR, DR may accelerate the progression of glaucoma. Severe types of glaucoma, such as neovascular glaucoma, can also significantly impact visual acuity. However, in this study, glaucoma was not classified in detail, and additional research on this topic is required.

This study has several limitations. First, it was based on presenting visual acuity; therefore, refractive errors might have influenced the assessment of VI. Second, the presence or absence of diseases was differentiated using claims code data; therefore, individual diagnoses may not have been accurate. Third, because the exact cause of VI could not be determined, further analyses were not feasible. Fourth, this study used data from 2015–2016, which are relatively outdated and may not reflect recent trends. Fifth, the NHIS data used in this study only provided information on the presence or absence of diseases, and there was no information on the severity of diseases that may affect visual acuity.

Using large-scale data, we analyzed the effects of major systemic adult diseases (such as HTN and DM) and major blindness-causing ocular diseases (such as DR and glaucoma) on VI. The role of each disease and the effects of various combinations of diseases were determined. Most of the results were similar to those of previous studies; however, in our study, glaucoma was negatively correlated with the risk of VI in the absence of DR. It was assumed that periodic ophthalmologic examinations for glaucoma, which mainly affects peripheral vision rather than central vision, were effective in preventing VI caused by other diseases. These findings provide evidence that regular eye examinations can prevent visual impairment.
